This article has been retracted.

# Effects of Omega-3 Polyunsaturated Fatty Acids on Cognitive Function after Splenectomy in Rats

**DOI:** 10.1155/2021/5513886

**Published:** 2021-12-26

**Authors:** Yong Guo, Feng Ping, Yongmei Cao, Jiawei Shang, Junfeng Zhang, Hong Jiang, Shudong Fang

**Affiliations:** ^1^Department of Critical Care Medicine, Shanghai Jiao Tong University Affiliated Sixth People's Hospital, Shanghai 200233, China; ^2^Department of Anesthesiology, Shanghai Jiao Tong University Affiliated Sixth People's Hospital, Shanghai 200233, China; ^3^Department of Anesthesiology, Shanghai Ninth People's Hospital, Shanghai Jiao Tong University School of Medicine, Shanghai 200011, China

## Abstract

**Background:**

Postoperative cognitive dysfunction (POCD) is a common complication after abdominal surgery. Several studies have reported that POCD is related to neuroinflammation caused by surgery. Omega-3 polyunsaturated fatty acids (PUFAs) can effectively inhibit the systematic inflammatory response. So, we use fish oil to study the effect of fish oil on inflammation, immunity, and cognitive behavior after splenectomy in rats.

**Methods:**

60 SD (Sprague-Dawley) rats were randomly divided into control group (group C, *n* = 20), surgery group (group S, *n* = 20), and omega-3 (fish oil) intervention group (group F, *n* = 20). Omega-3 PUFA was injected intraperitoneally from 3 days before operation to 7 days after operation in group F, and normal saline was injected simultaneously in group S. Rats in group S and group F received splenectomy under general anesthesia. Morris water maze behavioral evaluation was performed on the first, third, fifth, and seventh day after operation. The levels of IL-1*β* (interleukin-1*β*), IL-6 (interleukin-6), TNF-*α* (tumor necrosis factor-*α*), SOD (superoxide dismutase), and GSH-PX (glutathione peroxidase) were detected.

**Results:**

Serums IL-1*β*, IL-6, and TNF-*α* concentrations in group S and group F were higher than those in group C (*P* < 0.01), while those inflammatory cytokines in group F were significantly lower than those in group S (*P* < 0.01); serum GSH-PX levels in group F were higher than group S (*P* < 0.01). The Morris water maze behavior test performance of group F was better than that of group S (*P* < 0.05).

**Conclusion:**

Omega-3 PUFA can effectively improve postoperative inflammatory response, reduce the damage of antioxidant defense system, and improve postoperative cognitive function.

## 1. Introduction

Postoperative cognitive dysfunction (POCD) is a central nervous system (CNS) complication after anesthesia and surgery. Its clinical symptoms are memory loss, abstract thinking, and disorientation, accompanied by decreased social activities and fusion ability [1, 2]. POCD is common in surgical patients, which not only affects the quality of life of patients and increases the medical burden but also increases the incidence of postoperative complications and mortality of patients [3, 4]. Current studies suggest that the pathogenesis of POCD is not very clear. Low level of education, preoperative cognitive dysfunction, severe complications, long-term anesthesia, and secondary surgery are the key factors for POCD [5, 6]. At present, research on POCD mainly involves genes, surgery, trauma, stress, hypoxia, calcium homeostasis, inflammatory response, etc., and its pathogenesis mainly involves gene theory, epigenetic theory, neurotransmitter theory, brain injury theory, amyloid-*β* (a-*β*) theory, and neuroinflammation theory [7]. However, in recent years, a large number of studies have found that various mechanisms of POCD ultimately work through a common pathway—neuroinflammation. Some scholars believe that neuroinflammatory reaction is the central link in the occurrence and development of POCD and plays a key role in the occurrence and development of POCD [8].

Omega-3 polyunsaturated fatty acids (PUFA) (fish oil injection) can effectively inhibit the body's inflammatory response. The possible mechanism is that EPA (c20:5, omega-3) and DHA (c22:6, omega-3) in omega-3 polyunsaturated fatty acids family can replace arachidonic acid (AA, omega-6) in cell membrane phospholipids and compete for cyclooxygenase and lipoxygenase, thus reducing the inflammatory mediators from AA and reducing inflammation. So, we used PUFA to explore the effects of PUFA on postoperative inflammation, immunity, and cognitive behavior of rats.

## 2. Materials and Methods

### 2.1. Animal Model Preparation and Grouping

SPF (specific pathogen-free) male Sprague-Dawley (SD) rats weighing 200-250 g were purchased from Department of Experimental Animal Science, Shanghai Jiao Tong University (animal experiment ethics no: 2017-0268.). Sixty SD rats were randomly divided into the control group (group C, *n* = 20), operation group (group S, *n* = 20), and fish oil intervention group (group F, *n* = 20). In group F, omega-3 fish oil fat emulsion was injected intraperitoneally from 3 days before operation to 7 days after operation. In group S, normal saline was injected at the same time. Splenectomy was performed in groups S and F under 3% inhaled sevoflurane anesthesia. Behavioral examination and biological samples were collected during perioperative period. All biosafety procedures were approved by the experimental animal ethics committee of Shanghai Jiao Tong University.

### 2.2. Reagents and Instruments

Omega-3 fish oil fat emulsion injection (Omegaven®) was purchased from Fresenius Kabi Austria GmbH (Wuxi, China). The ELISA (enzyme-linked immunosorbent assay) kits for IL-1*β* (interleukin-1*β*), IL-6, and TNF-*α* (TNF-*α* (tumor necrosis factor-*α*)) were imported and repackaged (R&D Company, USA). Superoxide dismutase (SOD) and glutathione peroxidase (GSH-PX) kits were purchased from Nanjing Jiancheng Reagent Company.

### 2.3. Medication, Surgical Treatments, and Behavioral Tests

Group S and group F underwent open splenectomy. All the experimental rats were fasted on the day of surgery, and they started to feed normally 1 day after surgery. After 1-5 days after operation, group F was given intraperitoneal injection of fish oil (2 ml/kg) every day; group C and group S were given normal saline. The Morris water maze is used to detect and evaluate the learning and memory ability of rats, which is divided into two parts: (1) place navigation test (seconds) and (2) spatial probe test (frequency). Morris water maze behavioral tests were performed before surgery and on the first, third, fifth, and seventh day after surgery. At the same time, blood samples were collected.

The experimental rats were sacrificed 7 days after operation, and samples were taken for testing. The specific anesthesia surgery methods for splenectomy and perioperative behavioral tests refer to previous study [9].

### 2.4. Sample Preparation and Detection

1. Blood test: 2% sodium pentobarbital (0.35 ml/100 g) was injected subcutaneously into the abdomen. After anesthesia, the tail vein blood was collected, centrifuged at 3000 r/min, and IL-1B, IL-6, TNF-*α*, SOD, and GSH-PX were detected according to the kit instructions
2. Histological observation: First perfuse the living heart, open the chest cavity, insert the needle into the left ventricle, and then clamp it with hemostatic forceps. Then, cut the right atrial appendage, inject about 300 ml of normal saline within 2-4 minutes to replace the circulating blood, and then inject about 150 ml of 4% paraformaldehyde solution within 1-2 minutes for in vivo fixation. All perfusion solutions are precooled at 4°C. Then, the head was decapitated, the skull was opened, and the whole brain was removed. The coronal slices containing the hippocampus and striatum were cut with the aid of a stereotaxic device, fixed with 4% paraformaldehyde, washed with water at 4°C overnight, dehydrated with gradient alcohol, transparent xylene, embedded in paraffin, and sectioned. HE (hematoxylin-eosin) staining was used to observe the changes in cell morphology

### 2.5. Statistical Methods

SPSS 16.0 software was used to analyze the data. The data were expressed as mean ± standard deviation ($\overset{¯}{x}\pm s$). LSD (least significant difference) and *S*-*N*-*K* tests were used for comparison among different groups, and paired *t*-test was used for comparison at different time points in the same group. A *P* value of less than 0.05 was considered statistically significant.

## 3. Results

### 3.1. Morris Water Maze Test Results

As shown in Figures 1 and 2, there was no difference in the results of place navigation test and spatial probe test between groups before surgery (*P* > 0.05). After surgery, the results of place navigation test and spatial probe test of group C were better than those of group F and group S. Besides, the results of water maze test performance between group F and group S after surgery were different. The group F performed better than the group S in the water maze test (*P* < 0.01).

### 3.2. Measurement of Serum Biochemistry Indicators

As shown in Figures 3, 4, and 5, inflammatory factors IL-1*β*, IL-6, and TNF-*α* increased after surgery. Serum IL-1*β*, IL-6, and TNF-*α* concentrations in group S and group F were higher than those before surgery (*P* < 0.01), while those inflammatory cytokines in group F were significantly lower than those in group S (*P* < 0.01). As shown in Figures 6 and 7, the enzyme activity of SOD and levels of GSH-PX decreased after surgery. Serum enzyme activity of SOD and levels of GSH-PX in group F were higher than those in group S (*P* < 0.01).

### 3.3. Pathological Examination of Rat Hippocampus

As shown in Figures 8 and 9, the pathological HE staining of hippocampus and striatum showed that in group C, the neurons in the hippocampus and striatum were arranged compactly, with normal cell morphology and no obvious damage; in group S, the neurons were arranged sparsely, with normal cell morphology and visible cell contour, but the cytoplasmic staining became shallow, some cells had nucleolus shrinkage, and some cells had annular bands around them; in group F, the number of neurons in the hippocampus and striatum was higher than that in group S. There was a significant improvement. In addition, the striated cell bridge structure connecting putamen and caudate nucleus was clearly visible in group C and sparse and fuzzy in group S, and the above situation in group F was significantly improved more than that in group S.

## 4. Discussion

Our research results show that due to surgical trauma and stress, IL-1*β*, IL-6, and TNF-*α* are significantly increased after surgery, SOD and GSH-PX are significantly reduced after surgery, and behavioral tests in rat performance have also dropped significantly. By supplementing omega-3 PUFA during the perioperative period, the postoperative inflammation was alleviated and the behavioral performance of the rats was improved. In addition, through histopathological examination, it was found that supplementation of omega-3 PUFA during the perioperative period can protect the central neuron cells from stress damage caused by surgical trauma. Regarding the mechanism of action of omega-3 PUFA, we believe that, on the one hand, it can inhibit the expansion of the body's inflammatory response [10] and enhance the ability to resist oxidative stress; on the other hand, intraperitoneal injection may inhibit inflammatory signals locally.

POCD is a central nervous system complication after surgery, manifested as confusion, anxiety, personality changes, and memory impairment [1, 2]. The mechanism of POCD involves cerebrovascular disease, cerebral blood perfusion, preoperative cognitive impairment, genetic susceptibility, changes in neurotransmitter function, and central nervous system inflammation (with inflammatory mediators IL-1*β*, TNF-*α*, IL-6, and others) [6, 11, 12]. It is currently believed that POCD is induced by surgery and anesthesia on the basis of neurodegeneration and is the result of the synergistic effect of multiple factors. It may be related to the patient's own factors, such as age, mental factors, genetic factors, sleep disorders, combined underlying diseases, alcohol and smoking, and education level; perioperative factors such as type of surgery, anesthesia methods, anesthesia drugs and other drugs, depth of anesthesia, hypoxia, hypotension, postoperative infection, postoperative pain, secondary surgery, and many other factors are related [6, 13]. Multiple animal experiments have proved that the increase in proinflammatory cytokines caused by surgery is related to cognitive impairment and neurodegeneration [14–16]. Moreover, the stress response caused by surgery is related to POCD [17]. Our animal experiments found that the operation caused the increase of serum IL-1*β*, IL-6, and TNF-*α* and the decrease of SOD and GSH-PX. Histopathology found that the neuronal cells in the operation group were sparsely arranged, and the cell morphology was normal, but the cytoplasm was stained lightly, some cells shrank nucleoli, and some cells appeared ring-shaped bands around them. These changes suggest that surgery can cause systemic inflammation, damage the ability to resist oxidative stress, and cause histological changes in central neurons.

Metabolic disorders of polyunsaturated fatty acids (PUFAs) have been reported to be related to a variety of neurological diseases, such as depression, bipolar disorder, schizophrenia, attention deficit hyperactivity disorder, and Alzheimer's disease (AD) [18, 19]. Among them, omega-3 PUFAs (ALA, EPA, and DHA) play an important role in the process of neurogenesis, synaptic development, and synaptic plasticity [20, 21]. Dietary supplementation of polyunsaturated fatty acids (PUFAs), especially omega-3 PUFA, shows outstanding effects in antioxidant and immune regulation [22]. Studies have shown that long-chain omega-3 PUFAs can reduce the risky process of patients with high-risk schizophrenia [23]; large intake of omega-3 PUFAs is associated with low levels of *β*-amyloid 42 (A*β*42) in plasma [24]. The development of white matter hyperintensity was associated with a low serum EPA/AA ratio but was not related to a low serum DHA/AA ratio [25]. In the rat animal model of traumatic brain injury (TBI), intraperitoneal injection of omega-3 polyunsaturated fatty acids can reduce microglia-mediated nerves by inhibiting the HMGB1/TLR4/NF-*κ*B pathway inflammation [26]. A study just published in cells reported that oral linoleic acid can rescue C57BL/6N mice (8 weeks old) from neuroinflammation and cognitive dysfunction induced by *β*-amyloid peptide (intraventricular injection) [27]. Omega-3 PUFA can activate blood vessel cells, restore elasticity of blood vessels, and repair damaged blood vessel walls; at the same time, they can effectively reduce blood viscosity, accelerate blood circulation, and quickly regulate High-density lipoprotein, Low-density lipoprotein, Glycerol triester and Cholesterol. Therefore, omega-3 PUFAs also have the potential to prevent POCD. Our animal experiments have found that supplementation of omega-3 PUFA during the perioperative period can reduce postoperative inflammation, enhance the ability to resist oxidative stress, protect the structure of central neurons, and improve neurobehavioral performance.

In summary, the development of POCD may be associated with postoperative excessive inflammation and oxidative stress. Supplementing experimental rats with omega-3 PUFA during the perioperative period may reduce systemic inflammation, antagonize early postoperative oxidative stress, and improve POCD.

## Figures and Tables

**Figure 1:** The results of place navigation test of three groups. The results of group F were better than those in group S (*P* < 0.01). (a) *P* < 0.01, group S vs. C. (b) *P* < 0.01, group F vs. C. (c) *P* < 0.01, group F vs. S.

**Figure 2:** The results of spatial probe test of three groups. The results of group F were better than those in group S (*P* < 0.01). (a) *P* < 0.01, group S vs. C. (b) *P* < 0.01, group F vs. C. (c) *P* < 0.01, group F vs. S.

**Figure 3:** The kinetics of IL-1*β* during the perioperative period. (a) *P* < 0.01, group F vs. S.

**Figure 4:** The kinetics of IL-6 during the perioperative period. (a) *P* < 0.01, group F vs. S.

**Figure 5:** The kinetics of TNF-*α* during the perioperative period. (a) *P* < 0.01, group F vs. S.

**Figure 6:** The kinetics of SOD during the perioperative period. (a) *P* < 0.01, group F vs. S.

**Figure 7:** The kinetics of GSH-PX during the perioperative period. (a) *P* < 0.01, group F vs. S.

**Figure 8:** Pathological staining of the hippocampus (dentate gyrus) before and 7 days after operation (HE, ×200).

**Figure 9:** Pathological staining of the striatum before and 7 days after operation (HE, ×200).

## Data Availability

The data used to support the findings of this study are available from the corresponding authors upon request.
